# Beneficial Effects of the Genus *Aloe* on Wound Healing, Cell Proliferation, and Differentiation of Epidermal Keratinocytes

**DOI:** 10.1371/journal.pone.0164799

**Published:** 2016-10-13

**Authors:** Mariko Moriyama, Hiroyuki Moriyama, Junki Uda, Hirokazu Kubo, Yuka Nakajima, Arisa Goto, Junji Akaki, Ikuyo Yoshida, Nobuya Matsuoka, Takao Hayakawa

**Affiliations:** 1 Pharmaceutical Research and Technology Institute, Kindai University, Higashi-Osaka, Osaka, Japan; 2 Central R&D Laboratory, KOBAYASHI Pharmaceutical Co., Ltd., Ibaraki, Osaka, Japan; University of Alabama at Birmingham, UNITED STATES

## Abstract

*Aloe* has been used as a folk medicine because it has several important therapeutic properties. These include wound and burn healing, and *Aloe* is now used in a variety of commercially available topical medications for wound healing and skin care. However, its effects on epidermal keratinocytes remain largely unclear. Our data indicated that both *Aloe vera* gel (AVG) and Cape aloe extract (CAE) significantly improved wound healing in human primary epidermal keratinocytes (HPEKs) and a human skin equivalent model. In addition, flow cytometry analysis revealed that cell surface expressions of β1-, α6-, β4-integrin, and E-cadherin increased in HPEKs treated with AVG and CAE. These increases may contribute to cell migration and wound healing. Treatment with *Aloe* also resulted in significant changes in cell-cycle progression and in increases in cell number. *Aloe* increased gene expression of differentiation markers in HPEKs, suggesting roles for AVG and CAE in the improvement of keratinocyte function. Furthermore, human skin epidermal equivalents developed from HPEKs with medium containing *Aloe* were thicker than control equivalents, indicating the effectiveness of *Aloe* on enhancing epidermal development. Based on these results, both AVG and CAE have benefits in wound healing and in treatment of rough skin.

## Introduction

The genus *Alo*e comprises about 600 species [1], most of which are native to South Africa. It has been used for medicinal purposes for probably over 4000 years. However, only a few species of *Aloe*, including *Aloe vera* and Cape aloe, have been reported to contain many bioactive ingredients. These *Aloe* species are currently listed in the pharmacopeia of many countries as laxatives.

*Aloe vera* (*Aloe barbadensis* Miller) is native to the Mediterranean region of southern Europe and North Africa, and to the Canary Islands. It is commonly grown in Asia, southern Europe, southern USA, Mexico, Aruba, Bonaire, Bermuda, the Bahamas, the West Indies, and Central and South America. According to a famous legend, Alexander the Great, upon the advice of Aristotle, conquered the island of Socotra to secure supplies of *Aloe vera* in order to treat wounded soldiers. It has also been reported that Christopher Columbus used *Aloe vera* to treat injured crewmembers. In ancient Egypt, Queen Nefertiti and Queen Cleopatra used aloe gel as a beauty aid [2–4].

*Aloe vera* is the most commercialized of all *Aloe* species. *Aloe vera* gel (AVG) contains no barbaloin, a metabolite responsible for the strong laxative effect of *Aloe*. Therefore, AVG has been used as an ingredient in food products, and for the production of gel-containing health drinks and yogurt. In addition, it has been used as a base material for the production of creams, lotions, soaps, shampoos, facial cleansers, and other products in the cosmetic industry.

Cape aloe *(Aloe ferox* Miller, *Aloe africana* Miller, *Aloe spicata* Baker, and their hybrids) is widespread in the Eastern Cape province of South Africa. In contrast to the food and cosmetic industry applications of *Aloe vera*, Cape aloe is mainly used in the treatment of a variety of diseases including skin wound healing, burns, eczema, and psoriasis [5–7]. However, most claims regarding the medicinal properties of Cape aloe are based on historical use. There are few controlled scientific investigations into the epidermal effects of Cape aloe when compared with investigations into the effects of *Aloe vera*. This may be due to the strict control of international trade, by the Endangered Species of Wild Fauna and Flora treaty (CITES) [8], of almost all species of *Aloe*, excluding *Aloe vera*.

The epidermis, the outer layer of the skin, acts as a physical barrier against pathogens, toxins, and harmful irradiation. Barrier function of the skin is thought to be mainly due to the outermost cornified layer. As the cells in the inner layer, called the basal layer, differentiate, they move towards the skin surface from the basement membrane to the spinous layer, then to the granular layer, and finally they transform drastically into corneocytes in the cornified layer. It is well known that the gradient of calcium level in the epidermis, defined by its low content in the basal layer and the highest level in the cornified layer, induces keratinocyte differentiation and contributes to from proper epidermal barrier formation [9]. In order to restore the barrier function, wound healing is an extremely important furture of skin epidermis.

Despite being used in the skin-wound healing and cosmetic industries, the effects of AVG juice and Cape aloe leaf extract on epidermal keratinocytes have not been fully investigated. Most research investigating the effects of AVG and Cape aloe extract (CAE) on wound healing and skin repair have been conducted on animal models or in clinical trials [5–7]. Only a few studies indicating that AVG has a beneficial effect on the proliferation of keratinocytes have been conducted [10, 11].

Traditionally, whole leaves and roots of Cape aloe and the gel from the whole leaf of *Aloe vera* are applied topically to treat skin wounds, burn, eczema, dermatitis, and acne. Many active ingredients including vitamins, enzymes, minerals, sugars, lignin, salicylic acids, and amino acids have been identified from these species. However, therapeutic effects have not correlated well with each individual component. Recently, a study exploring the biological effects of a single component from *Aloe* species was conducted. Choi et al reported that a 5.5 kDa glycoprotein isolated from AVG by activity-guided sequential fractionation was found to enhance keratinocyte proliferation and migration, and thereby accelerate wound healing [11]. However, it is currently believed that biological activities associated with *Aloe* arise from the synergistic actions of multiple compounds rather than from a single component [12]. In light of this hypothesis, we considered it relevant to examine whether a whole-leaf extract of Cape aloe or AVG had effects on epidermal function.

In this study, we focused on the effects of AVG and CAE on human primary epidermal keratinocytes (HPEKs). Migration, proliferation, and differentiation potential of epidermal keratinocytes, which is indispensable for skin wound healing, was enhanced by AVG or CAE treatment. In addition, the effects of AVG and CAE on cell surface expression of the cell adhesion molecules, integrin and cadherin, were assessed. These cell adhesion molecules contribute to epidermal function. Finally, the effects of AVG and CAE on a construction of human epidermal equivalent model were evaluated. Overall, this cellular and molecular approach was designed to provide a scientific understanding of the effect of AVG and CAE on epidermal functions. This is important given the extensive use of *Aloe* products in the medical and cosmetics industry.

## Material and Methods

### Test substances

The AVG powder and the dried leaves of Cape aloe were prepared by Kobayashi Pharmaceutical Co., Ltd. (Osaka, Japan). To obtain CAE powder, the dried leaves were extracted twice with hot water for 2 h and then the aqueous extract was evaporated under reduced pressure and lyophilized. The concentrations of identified chemical constituents in AVG and CAE are presented in Table 1.

**Table 1:** Chemical constituents of AVG and CAE.

Components	AVG	CAE
	(mg/100 g of dry powder)	(mg/100 g of dry powder)
**Sugars (hydrolyzed)**		
glucose	13,700	20,600
mannose	9,800	ND^a^
galactose	300	900
**Minerals**		
calcium	5,990	5,220
magnesium	533	1,270
sodium	3,170	565
**Anthraquinones**		
barbaloin	ND^a^	267
isobarbaloin	ND^a^	271

^a^ Not detected

### Cell culture

HPEKs were purchased from CELLnTEC (Bern, Switzerland) and maintained in CnT-PR (CELLnTEC) culture medium according to the manufacturer's protocol. Human skin equivalents were generated using CnT-02-3DP culture medium (CELLnTEC) according to the manufacturer’s protocol.

### Scratch assay

HPEKs were seeded on a 12-well culture plate and grown to confluence. The cell monolayer was then scraped to create a scratch with a pipet tip. Wound closure was measured with the EVOS FL Auto time-lapse imaging system (Thermo Fisher Scientific, Waltham, MA, USA).

### Wound-healing assay

Human full-thickness skin equivalents (EpiDerm-FT) were purchased from MatTek Corporation (Ashland, MA, USA), and cultured at the air-liquid interface according to the manufacturer’s instructions. Superficial incisional wounds, in which only the epidermis was removed, were created using 3 mm biopsy punches. Wound healing was evaluated by histological analysis.

### Histology and immunofluorescent analysis

Skin equivalents were fixed in 4% paraformaldehyde, embedded in optimal cutting temperature (OCT) compound, frozen, and sectioned at 10 μm. Sections were then either subjected to hematoxylin and eosin staining or immunohistochemical analysis as previously described [13]. The following antibodies were used as primary antibodies: rabbit polyclonal antibody against Ki67 (1/250) (NOVUS Biological, Littleton, CO, USA), rabbit polyclonal antibody against p63 (1/200) (SantaCruz, Dallas, TX, USA), rabbit polyclonal antibody against loricrin (1/1000) (BioLegend, San Diego, CA, USA), and chick polyclonal antibody against Keratin 15 (1/1000) (BioLegend). Staining was performed using specific secondary antibodies conjugated to Alexa 488 or 546 (1/1000). 4',6-Diamidino-2-phenylindole (DAPI) (Dojindo, Tokyo, Japan) was used for nuclear staining.

### RNA extraction, cDNA generation, and quantitative polymerase chain reaction

Total RNA was extracted using the RNeasy Mini Kit (Qiagen, Hilden, Germany) according to the manufacturer’s instructions. cDNA was generated from 1 μg of total RNA using the Verso cDNA Synthesis Kit (Thermo Scientific) and purified using the MinElute PCR Purification Kit (Qiagen). Quantitative polymerase chain reaction (q-PCR) analysis was conducted using the SsoFast EvaGreen supermix (Bio-Rad, Hercules, CA, USA) according to the manufacturer’s protocols. The relative expression value for each gene was calculated using the ΔΔCt method, and the most reliable internal control gene was determined using geNorm Software (Biogazelle, Zwijnaarde, Belgium). Details of the primers used in these experiments are shown in Table 2.

**Table 2:** Primer pairs used in this study.

Gene	Primer sequence (5′-3′)
*UBC* F	ATTTGGGTCGCGGTTCTTG
*UBC* R	TGCCTTGACATTCTCGATGGT
*B2M* F	TATCCAGCGTACTCCAAAGA
*B2M* R	GACAAGTCTGAATGCTCCAC
*ACTB* F	CATGTACGTTGCTATCCAGGC
*ACTB* R	CTCCTTAATGTCACGCACGAT
*GAPDH* F	CATGAGAAGTATGACAACAGCCT
*GAPDH* R	AGTCCTTCCACGATACCAAAGT
*GUS* F	CACCAGGGACCATCCAATACC
*GUS* R	GGTTACTGCCCTTGACAGAGA
*H6PD* F	GGGGTCACAGTTTTAGCTTCC
*H6PD* R	CCGTCTTCAGTTGGCGGTA
*UBE2D2* F	TGGCAAGCTACAATAATGGGG
*UBE2D2* R	GGAGACCACTGTGATCGTAGA
*UBE4A* F	GTACTTGGGATTTCACAGGTTGC
*UBE4A* R	GGCTAGAACTTTGCTGAGCATC
*IVL* F	TCCTCCAGTCAATACCCATCAG
*IVL* R	GCAGTCATGTGCTTTTCCTCTTG
*SPRR1B* F	TTCACACCAGGACCAGTCAC
*SPRR1B* R	CAAGGCTGTTTCACCTGCT
*SPRR2A* F	TCTGCCTTGGAGAACCTGAT
*SPRR2A* R	ACATGGCTCTGGGCACTTT

### Cell cycle assay

HPEKs were treated with 10 μg/mL of AVG or CAE for 48 h. After treatment, 5-ethynyl-2′-deoxyuridine (EdU) labeling and cell cycle analyses were conducted using the Click-iT EdU Alexa Fluor 488 Flow Cytometry assay kit (Thermo Fisher Scientific), according to the manufacturer's instructions. FxCycle Far Red (Thermo Fisher Scientific) was used to stain cells for DNA content. Cells were analyzed by flow cytometry (ec800 cell analyzer, SONY, Tokyo, Japan). FlowJo (TreeStar Inc., Ashland, OR, USA) software was used for quantitative analysis.

### Cell proliferation assay

HPEKs were seeded on a 96-well plate and incubated for 24 h in a CO_2_ incubator. The cells were then treated with 10 μg/mL or 100 μg/mL AVG or CAE for 48 h. The cell proliferation assay was performed using cell counting kit-F (Dojindo) according to the manufacturer’s protocol. Fluorescence was measured with excitation at 490 nm and emission at 515 nm using a Synergy H4 microplate reader (BioTeK, Winooski, VT, USA).

### Flow cytometry analysis

HPEKs were harvested and re-suspended in staining buffer (PBS containing 1% BSA, 2 mM EDTA, and 0.01% sodium azide) at a density of 1×10^6^ cells/mL, incubated for 20 min with a phycoerythrin (PE)-conjugated antibody against CD29, CD104, an allophycocyanin (APC)-conjugated antibody against CD324, or a brilliant violet 421-conjugated antibody against CD49f (BioLegend). Nonspecific staining was assessed using relevant isotype controls. Dead cells were excluded using the Live/Dead Fixable Far Red Dead Cell Stain Kit (Life Technologies). FlowJo software was used for quantitative analysis.

### Western blot analysis

Cells were lysed with lysis buffer (20 mM Tris-HCl [pH8.0], 1% SDS, and 1 mM DTT). Blots were probed with a rat monoclonal antibody against E-cadherin (Clone ECCD-2), mouse monoclonal antibody against β1-integrin (Clone BV7) (Abcam, Cambridge, UK; ab7168), and mouse monoclonal antibody against Actin (Clone C4) (Merck-Millipore, Billerica, MA, USA; MAB1501). Horseradish peroxidase (HRP)-conjugated anti-mouse or rat IgG secondary antibody (Cell Signaling Technology; #7076, #7077) was used as a probe, and immunoreactive bands were visualized with the Immobilon Western Chemiluminescent HRP substrate (Merck-Millipore). The band intensity was measured using ImageJ software.

## Results

### AVG and CAE promote wound healing in epidermal keratinocytes

In order to evaluate whether AVG and CAE play a crucial role in wound healing and migration of keratinocytes, we performed the following assays. First, HPEKs were treated with 10 μg/mL of AVG or CAE; both treatments caused a significant increase in the migratory ability of HPEKs (Fig 1A). Next, 10 μg/mL of AVG or CAE was directly applied onto a superficial incisional wound in which only the epidermis had been removed from human full-thickness skin equivalents. In control skin equivalents, only 1 out of 4 incisional wounds recovered completely 3 days after wound creation. In contrast, migration of keratinocytes from the wound margin occurred earlier in the aloe treatments. Two out of 4 wounds treated with AVG, and 3 out of 4 wounds treated with CAE closed completely 3 days after wound creation (Fig 1B). These data indicated that AVG and CAE could induce wound healing in epidermal keratinocytes.

**Fig 1:** Influence of AVG and CAE on the wound healing in human epidermal keratinocytes. (A) HPEKs were treated with 10 μg/mL AVG or CAE, and subjected to the scratch wound healing assay over 8 h. White dotted lines indicate wound margins. The graph indicates the mean ± SEM values for wound closure rates of the group from 9 independent experiments. *P<0.05. (B) AVG or CAE (10 μg/mL) was directly applied onto a superficial incisional wound in which only the epidermis had been removed from human full-thickness skin equivalents and cultured at the air-liquid interface for 3 days. Representative images of hematoxylin and eosin staining of each group are shown. Arrowheads indicate wound margins.

### AVG and CAE promote keratinocyte proliferation

Cell proliferation is another critical factor in wound healing. Both AVG and CAE significantly stimulated HPEK proliferation 48 h after treatment (Fig 2A). Nuclear incorporation of EdU was then examined to evaluate rates of DNA synthesis in HPEKs directly. DNA contents were also measured to evaluate cell-cycle progression. In AVG- or CAE-treated cells, the numbers of S phase cells were significantly higher than those in the control cells (Fig 2B), indicating that AVG and CAE both promoted cell cycle progression in HPEKs.

**Fig 2:** Influence of AVG and CAE on the proliferation of human epidermal keratinocytes. (A) HPEKs were treated with AVG or CAE (10 μg/mL or 100 μg/mL) for 48 h, and subjected to the cell proliferation assay. The graphs indicate the mean ± SEM values for proliferation rate (fold increase over control) from 20 independent experiments. **P<0.01, *P<0.05. (B) HPEKs were treated with 10 μg/mL AVG or CAE for 12 h, and subjected to the EdU incorporation assay. The graphs indicate the mean ± SEM values for percentage of EdU-positive (EdU^+^) cells from 5 independent experiments. **P<0.01. (C, D) Human full-thickness skin equivalents were treated with 10 μg/mL AVG or CAE for 3 days, and subjected to immunofluorescent staining against Ki67 (C) and p63 (D). The blue signals indicate nuclear staining. The dotted lines indicate the boundary between the epidermis and the dermis. Scale bars, 50 μm.

Proliferation of epidermal keratinocytes around the wound margin in the human skin equivalent model was evaluated 3 days after treatment with AVG or CAE by fluorescent staining of Ki-67 and p63. Ki-67 is a cell proliferation marker and p63 is an important molecule for maintenance of keratinocyte proliferative capacity. As shown in Fig 2C and 2D, both AVG and CAE treatment enhanced the expression of Ki-67 and p63. This suggested that the *Aloe* treatments had promoted keratinocyte proliferation.

### AVG and CAE enhance the cell surface expression of adhesion molecules

It is well known that cadherin and integrin play an essential role in fundamental physiological and pathological processes, including wound healing. Therefore, we performed flow cytometry analysis in order to evaluate the cell surface expression of these proteins. When compared with the control cells, HPEKs treated with AVG or CAE expressed significantly higher levels of β1-integrin (CD29), α6-integrin (CD49f), β4-integrin (CD104), and E-cadherin (CD324) (Fig 3A). Intriguingly, q-PCR analysis revealed that mRNA expression levels of *ITGB1*, *ITGA6*, *ITGB4*, and *CDH1* were not altered in HPEKs treated with AVG or CAE (Fig 3B). In addition, protein expression levels of β1-integrin and E-cadherin were not affected by AVG or CAE (Fig 3C). These data suggested that both AVG and CAE upregulate the cell surface expression of β1-, α6-, β4-integrin, and E-cadherin in a transcription- and translation-independent manner.

**Fig 3:** Influence of AVG and CAE on the expression of adhesion molecules in human epidermal keratinocytes. (A-C) HPEKs were treated with 10 μg/mL AVG or CAE for 2 days, and subjected to flow cytometry analysis (A), q-PCR analysis (B), and western blot analysis (C). (A) Representative histograms are shown. The graphs indicate the mean ± SEM values for median fluorescent intensity (MFI) from 6 independent experiments. **P<0.01, *P<0.05. (B) The graphs indicate the mean ± SEM values for relative expression from 4 independent experiments. (C) The extracted proteins were immunoblotted with the indicated antibodies. Graphs indicate the relative band intensities as determined by ImageJ software and plotted as the means of 3 independent experiments.

### AVG and CAE promote keratinocytes differentiation

Data from several *in vivo* studies have revealed that topical application of AVG can promote keratinocyte differentiation [14], although more investigations will be required to address this issue. We therefore evaluated the effects of AVG and CAE on differentiation in HPEKs. Morphological changes were observed at concentrations greater than 1 mg/mL of AVG and CAE (Fig 4A). Q-PCR analysis revealed that AVG and CAE promoted the expression of differentiation markers of keratinocytes *SPRR2A*, *SPRR1B*, and *IVL*, only at higher concentrations (>100 μg/mL) (Fig 4B).

**Fig 4:** Influence of AVG and CAE on the differentiation in human epidermal keratinocytes. (A, B) HPEKs were treated with 0, 1, 10, 100, 1000, 2000 μg/mL AVG or CAE for 2 days. (A) Representative phase-contrast images of each group. Scale bars, 400 μm. (B) Gene expression levels of *SPRR2A*, *SPRR1B*, and *IVL* were quantified by q-PCR analysis. The graphs indicate the mean ± SEM values for relative expression from 5 independent experiments. **P<0.01, *P<0.05.

It has been reported that the differentiation process of keratinocytes is initiated when cells are “switched” to calcium concentrations above 0.1 mM (the calcium switch) [15, 16]. We therefore measured the calcium concentrations of the AVG and CAE samples. As shown in Table 1, AVG contained 5990 mg calcium/100 g of dry powder. This is equivalent to 0.149 mM when AVG is tested at 100 μg/mL. CAE contained 5220 mg calcium/100 g of dry powder. This is equivalent to 0.13 mM when CAE is tested at 100 μg/mL. These data suggested that AVG and CAE promoted keratinocyte differentiation through the action of calcium ions when these treatments were used at higher concentration (> 100 μg/mL).

### AVG and CAE are advantageous for epidermal development

In order to evaluate the effects of AVG and CAE on epidermal development, a human epidermal equivalent model was constructed in culture medium containing AVG or CAE. The staining pattern of keratin 15 and loricrin was not obviously changed when compared with that of the control (Fig 5B). However, we found that loricrin-positive granular layers were significantly thicker in AVG or CAE-treated epidermal skin equivalents (Fig 5B and 5C). In addition, hematoxylin and eosin staining revealed that the thickness of the entire epidermis was significantly enhanced in the human epidermal equivalent model treated with AVG or CAE (Fig 5A and 5C). These data indicated that applications of AVG and CAE facilitated epidermal development.

**Fig 5:** Influence of AVG and CAE on the epidermal development in human epidermal equivalents. HPEKs were treated with AVG or CAE (10 μg/mL or 100 μg/mL). Frozen sections of skin equivalent model were then subjected to hematoxylin and eosin (HE) staining (A) or immunofluorescent staining for loricrin (LOR, green) and keratin 15 (K15, red) (B). The blue signals indicate nuclear staining. Scale bars, 20 μm. (C) The graphs indicate the mean ± SEM values for thickness of the whole epidermis or granular layer of the skin equivalent in micrometers. N = 20. **P<0.01, *P<0.05.

## Discussion

*Aloe* has been used as folk medicine for skin wounds or burn healing. They also have applications in the cosmetic industry. Despite this, the effects of AVG and CAE on epidermal keratinocytes have not been investigated. In the present study, we applied molecular and cellular approaches to generate scientific data on the effects of AVG and CAE on epidermal keratinocytes. Results indicated that both AVG and CAE may exert beneficial effects on wound healing and treatment for rough skin. Our data revealed that AVG and CAE significantly improved wound healing in HEPK cells (Fig 1). We further demonstrated that this could be attributed to enhanced HEPK cell proliferation (Fig 2) as well as increased cell-surface expression of β1-, α6-, β4-integrin, and E-cadherin (Fig 3).

It has been reported that integrins, such as α6β4 and β1 integrin, have a crucial role in re-epithelialization during wound healing by facilitating migration and proliferation of keratinocytes [17]. The effects of E-cadherin on epidermal wound healing, however, have not been fully investigated. Deletion of E-cadherin in a mouse model prevents the formation of an epidermal barrier by regulating tight junctions [18]. Recently, E-cadherin has also been shown to be essential for sheet migration during wound healing in intestinal epithelial and gastric mucosal cells [19, 20].

In this study, we did not determine whether β1-, α6-, β4-integrin, and E-cadherin, upregulated by AVG and CAE treatment, contributed to facilitating migration and proliferation of keratinocytes. Further analyses such as knockdown experiments, or inhibitory experiments using neutralizing antibodies, will be required to solve this issue. It may also be relevant to investigate whether the 5.5 kDa glycoprotein isolated from AVG, shown to enhance keratinocyte proliferation and migration [11], could also contribute to upregulation of β1-, α6-, β4-integrin, and E-cadherin.

Calcium contained in AVG and CAE is one candidate for enabling the proliferation and differentiation of epidermal keratinocytes. In this study, we found that AVG and CAE promoted expression of keratinocyte differentiation markers only at high concentrations (Fig 4). In contrast, lower concentrations (100 μg/mL) significantly facilitated proliferation of epidermal keratinocytes in 2D culture and in a human skin equivalent during wound healing (Fig 2). It has been reported that increasing extracellular calcium levels above 0.1 mM *in vitro* can induce expression of several genes related to keratinocyte differentiation [15, 16].

Boyce et al. demonstrated that cell proliferation rates are gradually increased between 0.03 mM and 0.3 mM calcium [21]. AVG and CAE, when applied at 100 μg/mL in the present study, had calcium ion concentrations of 0.149 mM and 0.13 mM, respectively. As CnT-PR medium contains 0.07 mM calcium, the total concentration of calcium in AVG or CAE-containing medium would be around 0.2 mM. Our present data indicating enhanced proliferation and differentiation at 100 μg/mL AVG or CAE are thus consistent with previous reports. However, other components, such as the 5.5 kDa glycoprotein referred to above, may also affect the proliferation and differentiation of epidermal keratinocytes. Indeed, it is currently believed that the biological activities of *Aloe* arise as a result of the synergistic action of many bioactive compounds rather than as an effect of one single “magic bullet” [22].

It has been reported that topical application of AVG in a hydrophilic cream significantly resolved psoriasis when compared with the placebo control [14]. The authors suggested that the AVG cream inhibited psoriatic plaques by suppressing proliferation and stimulatory differentiation of epidermal keratinocytes. It is notable that the cream contained 0.5% (5 mg/mL) of AVG. Our data demonstrating that higher concentrations of AVG significantly promoted keratinocyte differentiation are therefore consistent with this earlier report. However, we cannot exclude the possibility that it is the known anti-inflammatory effects of AVG [23] that may most contribute to a cure for psoriasis. This is especially true as psoriasis is a hereditary disease elicited by chronic activation of cutaneous T cells.

Many of the beneficial effects of *Aloe* have been attributed to the polysaccharides and glycoproteins present in the pulp. Acemannan, a β-(1,4)-acetylpolymannan, has been identified as the main active ingredient in the inner leaf gel of *Aloe vera* [24]. Acemannan consists of a long chain polymer composed of glucose and mannose. It can reach a molecular weight of approximately 30 to 40 kDa or greater. Acemannan has been shown to have many biological activities including anti-cancer, anti-inflammatory, anti-microbial, cell proliferation, and wound healing effects [24–26]. Intriguingly, we could not detect mannose in CAE (Table 1), suggesting that the CAE used in our present study contained little, if any, acemannan.

The present data are consistent with previous reports that demonstrated that the monosaccharides released after hydrolysis of leaves of *Aloe ferox* were predominantly glucose and galactose, while those from AVG were mannose only [27]. It has been also reported that mannose-6-phosphate in *Aloe* has wound healing and anti-inflammatory effects in rats [28]. Of note, the 5.5 kDa *Aloe* glycoprotein demonstrated to improve proliferation and differentiation of epidermal keratinocytes, contains a high percentage of mannose [11].

Our data indicated a large difference in the concentrations of mannose and/or of mannose-containing components of AVG and CAE (Table 1). These components therefore unlikely contribute solely to the beneficial effects of *Aloe* observed in this study. However, we cannot exclude the possibility that a large difference in the concentration of mannose and/or mannose-containing components could affect the biological properties of *Aloe*. For example, in this study, AVG (high mannose) was more effective than CAE (no mannose detected) in accelerating cell proliferation (Fig 2A).

When compared with *Aloe vera*, only a few scientific studies of Cape aloe gel components and of beneficial effects of Cape aloe on epidermal cells have been reported [27, 29]. It would therefore be interesting to compare the biological efficacy and chemical characteristics of these two *Aloe* species. Such data would also provide a better understanding of basic principles underlying gel composition variability. This would have possible applications in both chemotaxonomy and in developing commercial quality control procedures for *Aloe* products, including CAE.

In summary, we provide the first demonstration that AVG and CAE have beneficial effects on cell proliferation, differentiation, development, and wound healing of epidermal keratinocytes. Compositional differences between these *Aloe* species were observed for some parameters. These should be further evaluated for their relevance to medicinal and cosmetic applications.
